The article "An Improved EMG-Driven Neuromusculoskeletal Model for Elbow Joint Muscle Torque Estimation" was published in 2021. Journal: Appl Bionics Biomech.

# An Improved EMG-Driven Neuromusculoskeletal Model for Elbow Joint Muscle Torque Estimation

**DOI:** 10.1155/2021/1985741

**Published:** 2021-10-31

**Authors:** Bingshan Hu, Haoran Tao, Hongrun Lu, Xiangxiang Zhao, Jiantao Yang, Hongliu Yu

**Affiliations:** ^1^Institute of Rehabilitation Engineering and Technology, University of Shanghai for Science and Technology, Shanghai 200093, China; ^2^Shanghai Engineering Research Center of Assistive Devices, Shanghai 200093, China; ^3^Department of Neurology, Changhai Hospital Affiliated to Second Military Medical University, Shanghai 200433, China

## Abstract

The accurate measurement of human joint torque is one of the research hotspots in the field of biomechanics. However, due to the complexity of human structure and muscle coordination in the process of movement, it is difficult to measure the torque of human joints in vivo directly. Based on the traditional elbow double-muscle musculoskeletal model, an improved elbow neuromusculoskeletal model is proposed to predict elbow muscle torque in this paper. The number of muscles in the improved model is more complete, and the geometric model is more in line with the physiological structure of the elbow. The simulation results show that the prediction results of the model are more accurate than those of the traditional double-muscle model. Compared with the elbow muscle torque simulated by OpenSim software, the Pearson correlation coefficient of the two shows a very strong correlation. One-way analysis of variance (ANOVA) showed no significant difference, indicating that the improved elbow neuromusculoskeletal model established in this paper can well predict elbow muscle torque.

## 1. Introduction

Human joint torque is one of the key reference indexes in rehabilitation evaluation and human-machine interaction. Joint torque can be applied to patient rehabilitation and athlete training, assessment, prosthetic and orthosis design and control, and so on. Especially in rehabilitation training, the estimation of joint torque can not only provide a basis for judging the degree of rehabilitation of patients but also help rehabilitation equipment to identify the movement intention of operators more accurately. Some researchers use the surface electromyogram (sEMG) signal of biceps brachii to estimate the exercise intensity of subjects and map it to the elbow torque and design the control strategy of the rehabilitation robot based on torque estimation [1–3]. Applying the estimation results of ankle torque based on sEMG to the sinusoidal trajectory tracking task of the ankle exoskeleton robot can help exoskeleton equipment achieve more natural movement [4]. However, due to the complexity of human structure and muscle coordination in the process of movement, it is difficult to measure the torque of human joints in vivo directly. Accurate prediction of human joint torque is one of the most challenging topics in the field of biomechanics [5].

There are two main methods to solve the joint torque. One is to construct the inverse dynamic model of the human body. Pontonnier and Dumont proposed a method to obtain muscle force according to the captured human motion data and established a human inverse dynamic model [6]. Obusek et al., combined with the motion law of the mass center of the human upper limb, established the spring simple pendulum model and then solved the joint torque of the human ankle [7]. Due to the high dependence on the accuracy of the dynamic model, it is difficult for the above method to provide high-accuracy joint torque solution results. The second method is the prediction of joint muscle strength with sEMG signal as input. The second method can predict muscle force, reflect antagonistic muscle actuating, and reflect more abundant information of human movement and muscle activation. Therefore, in recent years, many scholars have proposed the method of using sEMG signals to solve joint torque, which has been used in human upper limb elbow joint [8], index finger [9], lower limb knee joint [10], and ankle joint [4].

There are two kinds of estimation methods for predicting the joint torque by EMG signal. One method is to establish a regression model between sEMG and joint torque by using the machine learning method, which is usually called “black box method.” The commonly used machine learning methods include neural network, linear classifier, and support vector machine. Peng et al. established two three-layer reverse BP neural network models to estimate the torque of hip and knee joints [11]. Meng et al. used the root mean square characteristics of sEMG signals of four lower limb muscles as the input of the support vector regression model to estimate human-robot interaction force [12]. The modeling process of the “black box method” is simple, but the establishment of the model depends greatly on the training samples. When the test samples are greatly different from the training samples, the estimation accuracy will be very unsatisfactory. In addition, when complex multijoint and multidegree of freedom motion is carried out, the complexity of the mapping model will increase greatly. Because the increase of training samples is usually very limited compared with the complexity of the sEMG model, it is difficult for the black box method to obtain satisfactory generalization performance.

That limitation can be overcome through the dynamic modeling of the neuromuscular and skeletal systems [13]. Chen et al. used the musculoskeletal biomechanical model to estimate the knee torque and verified the accuracy and availability of the model through the experimental results of 8 subjects at different walking speeds [14]. Hou et al. established the elbow neuromusculoskeletal model to estimate the joint torque during flexion and extension [15]. Joint torque prediction based on musculoskeletal model needs to collect a large number of motion parameters and human physiological parameters, and the process of muscle strength estimation is complex [1]. To meet the practical needs, it is necessary to simplify and optimize the musculoskeletal model. For example, the common dual-muscle musculoskeletal model is often used to predict the muscle torque of the elbow [16]. Linear optimization [17], genetic algorithm [18], nonlinear least squares optimization [19], and other methods are usually used to optimize the parameters in the musculoskeletal model for more accurate prediction.

Elbow joint and its accessory muscles play an important role in the movement of the upper limbs. The bone structure of the elbow joint is relatively simple, but it involves a large number of muscles. The commonly used elbow muscle bone model is the double-muscle model, which uses two muscle force lines to represent the biceps and triceps. The bone structure involved in the elbow is regarded as a connecting rod, and the radius of the upper arm and forearm is ignored in the calculation [20]. The model can quickly solve the muscle force, arm, real-time muscle fiber length, and muscle contraction speed according to the real-time joint angle, combined with sEMG signal and Hill muscle model, and then quickly obtain the muscle torque of elbow joint. However, the triangular relationship of triceps brachii is inconsistent with the physiological structure of the elbow joint. This will cause deviations in the calculation and then lead to a large error in the calculation result of the resultant torque. This paper discusses an improved elbow neuromusculoskeletal model. Based on the traditional double-muscle model, the biceps brachii muscle force is divided into two muscles, the triceps brachii muscle is divided into three muscles, and the brachialis is added as the flexor. The humeral trochlear was also taken into account. The improved model has more complete muscle quantity; the geometric model is more in line with the physiological structure and can predict the elbow muscle torque more accurately.

The rest of this paper is organized as follows: Section 2 introduces the physiological of the elbow joint; Section 3 introduces the optimization results of the main parameters of the elbow neuromusculoskeletal model; in Section 4, the elbow neuromusculoskeletal model proposed in this paper is used to predict the elbow muscle torque and compared with the simulation results of OpenSim software.  Section 5 is the conclusion of this paper.

## 2. Elbow Musculoskeletal Model

The elbow physical model is the basis of elbow muscle torque prediction. The elbow physiological model established in this paper includes three parts: Hill musculotendon model, elbow musculoskeletal model, and elbow joint kinematic and moment model. The Hill musculotendon model is used to calculate the force of muscle contraction according to muscle activation. The elbow musculoskeletal model consists of an amalgamation of muscle architecture and bone structure of the elbow joint. The elbow joint kinematic and moment model is used to determine the force arm of the elbow flexor and extensor groups acting on the rotation axis of the elbow joint during movement and finally solve the muscle resultant moment.

### 2.1. Hill Musculotendon Model

The improved Hill Musculotendon model shown in Figure 1 is generally used to solve the muscle contraction force [21]. The muscle model mainly includes series elastic element (see), passive elastic element (PEE), contraction element (CE), viscous damping element (VE), and pennation angle *φ* (in the following formulas, “CE,” “PE,” and “ve” are used as subscripts for the latter three, respectively). In Figure 1, *l*_mt_ is the length of muscle, *l*_m_ is the length of muscle fiber, and *l*_t1_ and *l*_t2_ are the length of tendon at both ends, respectively.

According to the Hill muscle model, the relationship between muscle length, muscle fiber length, and tendon length is as follows:

(1) $$\begin{array}{c} l_{\text{mt}}=l_{\text{m}}\cdot \cos\varphi +l_{t}=lE\cdot \cos\varphi +l_{\text{t}1}+l_{\text{t}2}. \end{array}$$

The muscle force is calculated as follows:

(2) $$\begin{array}{c} F_{\text{M}}=\left(F_{\text{CE}}+F_{\text{PE}}+F_{\text{VE}}\right)\cdot \cos\varphi . \end{array}$$

In equation (2), *F*_CE_, *F*_PE_, and *F*_VE_ are muscle fiber active force, muscle fiber passive force, and viscous damping force, respectively. *F*_VE_ is very small and is not considered in this paper. *F*_CE_ is determined by muscle activation, muscle fiber length, muscle fiber contraction speed, and maximum muscle strength. The calculation formula of *F*_CE_ is as follows:

(3) $$\begin{array}{c} F_{\text{CE}}=a\cdot f_{\text{l}}\cdot f_{\text{v}}\cdot F_{0}=f_{\text{CE}}\cdot F_{0}. \end{array}$$

In equation (3), *a*, *f*_l_, *f*_*v*_, and *F*_0_ are muscle activation, muscle fiber length influencing factor, muscle fiber contraction speed influencing factor, and resting maximum isometric contraction force, respectively. In equation (3), muscle activation *a* is calculated by the following formula [22]:

(4) $$\begin{array}{c} a\left(t\right)=\frac{e^{Au\left(t\right)}‐1}{e^{A}-1}. \end{array}$$

In equation (4), *a*(*t*), *u*(*t*), and *A* are muscle activation, normalized sEMG signal, and nonlinearity, respectively. The influence factor of muscle fiber length *f*_l_ and the influence factor of muscle fiber contraction speed *f*_*v*_ in equation (3) are calculated by the Thelen model [23], as shown in the following equation:

(5) $$\begin{array}{c} f_{\text{l}}=e^{-\left({\left(l_{\text{m}}/l_{\text{mopt}}-1\right)}^{2}/\gamma \right)}. \end{array}$$

In formula (5), *l*_m_ and *l*_mopt_ are the current muscle fiber length and resting muscle fiber length, respectively. *γ* is the shape factor. The calculation formula of *f*_v_ in equation (3) is

(6) $$\begin{array}{c} f_{\text{v}}=\left\{\begin{array}{cc} \frac{1+v_{\text{n}}}{1-\left(v_{\text{n}}/A_{\text{s}}\right)}, & v_{\text{n}}\leq 0,\\ \frac{f_{\text{M}}\cdot v_{\text{n}}+\left(\left(A_{\text{s}}\cdot \left(f_{\text{M}}-1\right)\right)/\left(2+2\cdot A_{\text{s}}\right)\right)}{v_{\text{n}}+\left(\left(A_{\text{s}}\cdot \left(f_{\text{M}}-1\right)\right)/\left(2+2\cdot A_{\text{s}}\right)\right)}, & v_{\text{n}}>0. \end{array}\right. \end{array}$$

In equation (6), *v*_n_ is the normalized contraction velocity; *A*_s_ is the curve parameter, taken as 0.25; and *f*_M_ is the maximum muscle force during muscle fiber elongation (normalizing the muscle fiber active force). The passive force *F*_PE_ can be calculated by the passive coefficient *f*_PE_ and the maximum muscle force *F*_0_, that is,

(7) $$\begin{array}{c} F_{\text{PE}}=f_{\text{PE}}\cdot F_{0}. \end{array}$$

*f*_PE_ can be calculated by muscle fiber length. When the length of muscle fiber is less than or equal to the resting length, no passive force will be generated. When the length of muscle fiber is greater than the resting length, a passive force will be generated. Thelen's formula is also used here [23]:

(8) $$\begin{array}{c} f_{\text{PE}}=\frac{e^{\left(k^{\text{PE}}\left(l_{\text{m}}/l_{\text{mopt}}-1\right)\right)/\varepsilon_{0}^{\text{M}}}-1}{e^{k^{\text{PE}}}-1}. \end{array}$$

In equation (8), *k*^PE^ is the curve shape parameter; *ε*_0_^M^ the maximum passive muscle tension strain. The pennation angle *φ* can be calculated as follows:

(9) $$\begin{array}{c} \varphi =\arcsin\left(\frac{l_{\text{mopt}}\sin\varphi_{0}}{l_{\text{m}}}\right). \end{array}$$

In equation (9), *φ*_0_ is the pennation angle corresponding to the resting length of muscle fiber *l*_mopt_, *φ* is the pennation angle corresponding to the muscle fiber length *l*_m_, and *w* is the muscle fiber width.

To sum up, the process of calculating muscle force using Hill musculotendon model is shown in Figure 2. The inputs to the model are real-time muscle fiber length *l*_m_ and real-time tendon length *l*_t_ (the calculation methods of *l*_m_ and *l*_t_ will be introduced in Section 2.3). The cosine value of pennation angle can be obtained from *l*_m_ according to equation (9). The normalized muscle fiber contraction velocity *v*_n_ can be obtained by deriving *l*_m_. By *l*_m_, cos *φ*, and *l*_t_, the real-time muscle length *l*_mt_ can be obtained according to equation (1). The influence factor of muscle fiber length *f*_l_ can be obtained from *l*_m_ according equation (5). The influence factor of muscle fiber speed *f*_v_ can be obtained from *v*_n_ according to equation (6). According to *a*_1_, *f*_l_, and *f*_v_, the active coefficient *f*_CE_ can be obtained according to equation (3). The passive coefficient *f*_PE_ can be obtained from *l*_mt_ according to equation (8). Summing *f*_CE_ and *f*_PE_ and multiplying by the cosine value of the pennation angle *φ* and the maximum muscle strength of muscle fiber *F*_0_ according to equation (2), the muscle strength *F*_M_ is obtained finally.

### 2.2. Elbow Physiological Model

The bone structure of the elbow joint is relatively simple, but it involves a large number of muscles, so it needs to be simplified. In the process of elbow flexion, the joint torque produced by the brachialis, the long head of biceps brachii, and short head of biceps brachii is large, and they are the main flexion muscles. It can be seen from the muscle force data of upper limb in reference [24] that, although the average force arm of the brachioradialis muscle is large, its peak force is relatively small. At the same time, according to the data in reference [25], the elbow torque provided by the brachioradialis muscle is smaller than that of the biceps brachii muscle and brachialis. Considering comprehensively, the brachioradialis muscle was not added in order to simplify the model in this paper. The elbow extensor muscle group mainly includes the triceps brachii and anconeus muscle. The maximum cross-sectional area of the anconeus muscle is relatively small, the muscle contraction force is also small, and the torque of the elbow joint is limited. In addition, this paper only establishes a two-dimensional musculoskeletal model of elbow flexion/extension in the sagittal plane to predict elbow muscle torque. The reasons are as follows: firstly, the three-dimensional elbow musculoskeletal model increases the number of parameters to be input in the model furtherly, which increases the complexity of the musculoskeletal model. Secondly, according to the motor anatomy of the human upper limb, the elbow joint is a natural hinge joint, which has only one degree of freedom of flexion/extension. In the process of flexion and extension, the relevant muscle forces are mainly used to make the elbow flexion and extension when excluding the influence of double-joint muscles.

Figure 3 shows the comparison of two-dimensional elbow musculoskeletal models, in which Figure 3(a) shows the commonly used elbow model [20]. The model uses two tension lines to represent the biceps brachii and triceps brachii. The bone structure involved in the elbow joint is regarded as a connecting rod, and the radii of the upper arm and forearm are ignored in the calculation. The model takes the rotation center of the elbow joint as the origin *O* and establishes a spatial rectangular coordinate system *O*-*xyz*. *Thex*-axis is parallel to the sagittal axis, and the direction is forward. The *y*-axis is parallel to the frontal axis and the direction points to the inner side of the body of the right hand. The *z*-axis is parallel to the vertical axis, and the direction is upward. The upper arm coincides with the *z*-axis and does not move vertically. The forearm rotates around the *y-*axis. *A* is the starting point of biceps brachii, *B* is the stop point of biceps brachii, and *C* is the position of *B* after elbow flexion. *D* is the starting point of triceps brachii, *E* is the ending point of triceps brachii, and *F* is the position of *E* after rotation; *θ* is the elbow flexion angle. *F*_Bi_ represents biceps brachii muscle strength, and *F*_Tr_ represents triceps brachii muscle strength.

It can be seen from Figure 3(a) that the geometric relationship between the starting and ending points of muscle and bone can be considered a triangular relationship, that is, the triangular *ODF* and triangular *OAC*.  Figure 4 shows a sagittal view of the humeral ulnar joint during flexion, in which the ending point of the flexor muscle group in the forearm bone is far from the rotation center. Therefore, the relationship between the muscle force line of the flexion muscle group and the bone during flexion can be calculated according to the triangular relationship. However, the ending point of extensor muscle group is located on the olecranon process of the ulna. When the ulna moves around the humeral pulley, the contraction trajectory of the extensor muscle is approximately a circular arc, which is different from Figure 3(a). Some scholars have improved the musculoskeletal model in Figure 3(a) according to the real anatomical structure of the elbow joints, as shown in Figure 3(b) [26]. The triceps brachii ending point *E* in Figure 3(b) is located on the red circle, which represents the humeral trochlea. When the extensor muscle contracts, its ending point moves around the arc, which is more in line with the physiological structure of the elbow.

In this paper, the model in Figure 3(b) is further improved to obtain the elbow musculoskeletal model shown in Figure 5. Firstly, in the musculoskeletal model of this paper, the two heads of the biceps brachii are divided into two muscles, the triceps brachii is divided into three muscles, and the brachialis is added as the flexor. Secondly, because the long head of the triceps brachii and biceps brachii is double-joint muscles that span the shoulder joint and elbow joint, part of the length is located on the shoulder joint, which is not within the triangular relationship, and considering the structure of the humeral trochlear, the starting and ending points of the main muscles in the elbow joint musculoskeletal model are considered in detail in this paper. The long head of triceps brachii is a double-joint muscle, so point *J* is set as the starting point of the long head of triceps brachii. The lateral head and medial head of triceps brachii are single joint muscles, the starting point is set at *D*_0_ and *D*_1_, and all ending points of the three heads of triceps brachii are *E*. When the upper arm is vertically stationary, due to the humeral trochlear structure, the ending points of triceps brachii change according to the arc track. Therefore, the change of *D*_0_, *D*_1_, *E*, and *J* points does not affect the calculation of the length of triceps brachii. They are set here to explain the structural characteristics of triceps brachii. The long head and short head of the biceps brachii are double-joint muscles that span the shoulder joint and elbow joint. Part of the length is located on the shoulder joint and is not within the triangular relationship. Based on the existing data analysis, the starting points of the two heads of biceps brachii are the same in the sagittal plane, but the activation degree is different during flexion. Set the starting point of both heads of the biceps brachii as *A*_0_, and the part crossing the shoulder joint is *A*_0_*A* segment. When the shoulder joint is not moving, the length of *A*_0_*A* segment remains unchanged. According to the anatomical characteristics of the brachialis, the *GH* segment is newly added as the path of the brachialis (when the elbow joint is in the extended position). In Figure 5, the position of the brachialis ending point *H* after rotation is point *I*. The specific position of the above starting and ending points is determined according to the anatomical data. In Figure 5, *F*_Bilong_, *F*_Bishort_, *F*_Bra_, *F*_Trlong_, *F*_Trlat_, and *F*_Trmed_ represent the muscle forces of the long head of biceps brachii, the short head of biceps brachii, the brachialis, the long head of triceps brachii, the lateral head of triceps brachii, and the medial head of triceps brachii, respectively.

### 2.3. Elbow Joint Kinematic and Moment Model

The main function of the elbow joint kinematic and moment model is to calculate the real-time muscle fiber length *l*_m_, real-time tendon length *l*_t_ and real-time muscle force arm *r*_m_ according to the joint flexion angle *θ* and elbow physiological model. Then, combined with the Hill muscle model, the muscle force *F*_M_ and the muscle torque acting on the elbow can be obtained. In this section, the long head of biceps brachii is taken as an example to introduce the calculation method of muscle force arm and the length of flexion muscle group. The short head of biceps brachii and brachialis can refer to this calculation method. Then, taking the long head of triceps brachii as an example, the calculation of muscle force arm and the length of extensor muscle group is introduced. Since the ending points of triceps brachii are located on the humeral trochlea and the force arm is almost constant, the medial head and lateral head of triceps brachii can refer to this calculation method.

For the long head of biceps brachii, if the coordinates of the starting point *A*, the ending point *B*, and the position *C* after the rotation of *B* are (*x*_1_, *y*_1_, *z*_1_), (*x*_2_, *y*_2_, *z*_2_), and (*x*_2_, *y*_2_, *z*_2_), there is the following transformation equation:

(10) $$\begin{array}{c} \overset{⟶}{OC}=R\overset{⟶}{OB},\\ R=\left[\begin{array}{ccc} \cos\theta & 0 & -\sin\theta \\ 0 & 1 & 0\\ \sin\theta & 0 & \cos\theta \end{array}\right]. \end{array}$$

In equation (10), $\overset{⟶}{OC}$ and $\overset{⟶}{OB}$ are the directed vectors from the origin *O* to point *C* and point *B*, respectively. *R* is the transformation matrix; *θ* is the elbow flexion angle.

The coordinates of point *C* can be obtained according to $\overset{⟶}{OC}$. The muscle length *l*_mtBi_ of the long head of biceps brachii after joint rotation is calculated as follows:

(11) $$\begin{array}{c} l_{\text{mtBi}}=\sqrt{{\left(x_{3}-x_{1}\right)}^{2}+{\left({\text{y}}_{3}-y_{1}\right)}^{2}+{\left(z_{3}-z_{1}\right)}^{2}}+l_{0}. \end{array}$$

In equation (11), *l*_0_ is the muscle length that does not belong to the triangular relationship. For the long head and short head of biceps brachii, it refers to segment *AA*_0_ in Figure 5. The real-time length *l*_mBi_ of muscle fiber can be obtained by subtracting the tendon length *l*_tBi_ from the muscle length *l*_mtBi_ of the long head of the biceps brachii. The change of tendon length *l*_tBi_ is very small. In this paper, it is treated as 1.02 times of resting tendon length *l*_toptBi_.

(12) $$\begin{array}{c} l_{\text{mBi}}=l_{\text{mtBi}}-l_{\text{tBi}}=l_{\text{mtBi}}-1.02\cdot l_{\text{toptBi}}. \end{array}$$

In this paper, the flexion motion is regarded as carried out in the sagittal plane, that is, the *xOz* plane. Then, the calculation formula of the force arm of the long head of biceps brachii *r*_Bi_ can be obtained according to the distance from the origin to the straight line in the two-dimensional plane:

(13) $$\begin{array}{c} \left\{\begin{array}{c} r_{\text{Bi}}=\frac{\left|b\right|}{\sqrt{k^{2}+1}},\\ b=-k\cdot x_{1}+z_{1},\\ k=\frac{z_{3}-z_{1}}{x_{3}-x_{1}}. \end{array}\right. \end{array}$$

For the long head of triceps brachii, Pigeon and Feldman found that the forced arm of this muscle increased slightly during extension [27]. In this paper, its treatment is as follows:

(14) $$\begin{array}{c} r_{\text{Tri}}=r_{0}-k_{\text{s}}\cdot \frac{\theta }{90}. \end{array}$$

In equation (14), *r*_0_ and *k*_s_ are the initial force arm value and shape parameters when the elbow joint is in the extended position. Because the ending points of the three muscles of the triceps brachii converge on the total tendon of the olecranon process, the force arms of the three muscles are always the same. The muscle length of the long head of triceps brachii *l*_mtTri_ is calculated as follows:

(15) $$\begin{array}{c} l_{\text{mtTri}}=\frac{l_{\text{moptTri}}+\theta \cdot r_{\text{Tri}}}{180}. \end{array}$$

The tendon length of the long head of triceps brachii is treated in the same way as equation (12). The real-time muscle fiber length *l*_mTri_ can be obtained by subtracting the tendon length *l*_tTri_ from the muscle length.

From equations (10)–(15), the muscle fiber length and muscle force arm of each muscle contained in the elbow muscle bone model in this paper can be obtained. Combined with the sEMG data of each muscle, the muscle force *F*_M_ of each muscle can be obtained according to the Hill muscle model in Section 2.1. The calculation formula of elbow muscle resultant moment is as follows:

(16) $$\begin{array}{c} \tau_{\text{human}‐\text{el}}\left(\theta ,t\right)=\overset{m}{\underset{i=1}{\sum }}\left(r_{i}\left(\theta \right)\cdot F_{\text{M}}^{i}\left(\theta ,t\right)\right.. \end{array}$$

In equation (16), *τ*_human−el_ represents the elbow muscle resultant moment when the joint angle is *θ* and the sampling time is *t*. *r*_*i*_(*θ*) is the *i*th muscle force arm when joint angle is *θ*. *F*_M_^*i*^(*θ*, *t*) is the *i*th muscle force when the joint angle is *θ*.

To sum up, the workflow of solving muscle torque by using the elbow musculoskeletal model is shown in Figure 6. Firstly, the sEMG_1_ signal of the first muscle in this model is processed to obtain the muscle activation *a*_*i*_. Then, according to the measured elbow flexion angle *θ*, the forward kinematics analysis is carried out. The real-time muscle fiber length *l*_m1_, real-time tendon length *l*_t1_, and real-time muscle force arm *r*_1_ were obtained. According to the Hill muscle model mentioned in Section 2.1, the muscle strength *F*_M_^1^ of the first muscle can be obtained. According to equation (16), the muscle force *F*_M_^1^ of the first muscle is multiplied by *r*_1_ to obtain the muscle torque *τ*_1_ of the first muscle acting on the elbow joint. Just like the first muscle, according to the joint flexion angle *θ* and the other muscle's surface EMG signals, the muscle torque can be obtained, respectively. By summing these moments, we can get the muscle torque *τ*_sum_ acting on the elbow joint.

## 3. Parameter Values in the Musculoskeletal Model

According to the analysis in the previous section, there are a large number of parameters to be input in the elbow musculoskeletal model. These parameters can be divided into two categories: formula parameters and personalized parameters. Formula parameters refer to widely verified and generalized parameters, such as shape parameters. The values of formula parameters in the musculoskeletal model in Section 2 are shown in Table 1.

Personalized parameters refer to the physiological and anatomical parameters of the calculated object, which may change due to different objects, including muscle activation, muscle fiber resting length *l*_mopt_, tendon resting length *l*_topt_, maximum muscle force *F*_0_, and resting pinnate angle *φ*_0_ and muscle space coordinate values. Muscle activation *A* is obtained by processing sEMG, which has been introduced in the workflow of the musculoskeletal model. In this paper, the sEMG signals of relevant muscles are not actually collected to obtain the activation degree but obtained by using the open source human musculoskeletal system simulation software OpenSim. Other personalization parameters as shown in Table 2 are obtained from the literature [24]. For different individuals, the resting length of muscle fibers and tendons can be scaled by height, and the maximum muscle strength needs to be measured.

In addition, the calculation of muscle fiber length of the flexion muscle group also requires muscle spatial coordinates (not required for extensor muscle group calculation). These data can be fitted in OpenSim through the muscle-related parameters in Table 2. For individual parameters of different heights, the scaling fitting method can be used. As shown in Table 3, the spatial parameters of the flexion muscle group are shown. For biceps brachii, the starting point and ending point in the table refer to the point *A* in the model in Figure 5, rather than the anatomical starting and ending point *A*_0_.

## 4. Simulation and Results

### 4.1. Simulation Setup

The musculoskeletal model in Section 2 is implemented in the numerical simulation software. To verify the elbow muscle torque prediction model proposed in this paper, the elbow angle data and the muscle activation of the six muscles contained in the musculoskeletal model need to be input. The elbow input angle of the model is shown in Figure 7. The elbow angle moves from 0° to 90° and then returns to 0° within 2 s, representing the flexion and extension movement of the elbow. OpenSim4.1 was used to calculate the main muscle force, muscle activation, and elbow muscle torque of the upper limb under the same exercise state. The extracted muscle activation is input into the numerical model, and the muscle force and elbow muscle torque calculated by the numerical model are compared with the results calculated by OpenSim.

The model used in OpenSim simulation is Arm26, which is an OpenSim self-contained upper limb musculoskeletal model. The right upper limb muscles introduced by the model include the long head of biceps brachii, the short head of biceps brachii, the long head of triceps brachii, the lateral head of triceps brachii, and the medial head of triceps brachii. Secondly, to prevent the influence of shoulder and elbow double-joint muscles on the prediction of elbow muscle torque, the shoulder joint was set as fixed after deenabling.

According to the elbow flexion and extension movement planned in Figure 7, the elbow forward kinematics, dynamics, and muscle activation data can be obtained according to the joint angle by using the Computed Muscle Control (CMC) function of OpenSim software. The activation range in OpenSim model is 0-1, but in order to make the model run normally, the activation is set to a number slightly higher than 0 by default, and this study is set to 0.02-1. The muscle activation derived from OpenSim fluctuates greatly before the end of muscle movement and needs smoothing. As shown in Figure 8, the muscle activation data obtained by the above method will be substituted into the numerical calculation model as one of the signal sources.

### 4.2. Simulation Results and Discussion

Using the elbow musculoskeletal model established in this paper, the muscle force time relationship and muscle length time relationship of relevant muscles are calculated and compared with the calculation results of OpenSim software (Figures 9 and 10).

Next, the curves in Figures 9 and 10 are analyzed from the perspective of Pearson correlation coefficient and one-way ANOVA. Pearson correlation is a method to measure correlation. One-way ANOVA can compare the differences between the two. The comparative analysis results of muscle force time relationship are shown in Table 4. According to Pearson correlation coefficient, the model results established by OpenSim and this study are an extremely strong correlation (ESC); that is, the change trend of the two is consistent, which is consistent with that in Figure 9. According to the results of one-way ANOVA, there was no significant difference (NSD) in the comparison results of the long head of biceps brachii, the long head of triceps brachii, and the lateral head of triceps brachii, but there was an extremely significant difference (ESD) among the brachialis, the short head of biceps brachii, and the medial head of triceps brachii. As can be seen from Figure 9, the three muscles are inconsistent with the OpenSim simulation results in some sections, indicating that there are some differences in the model. Since the formula parameters in the two models are the same, the main source of error is the above muscle personalized parameters, mainly the error of the coordinates of the starting and ending points of muscle anatomy.

Compare the muscle length-time relationship predicted by the OpenSim model and numerical model, and the results are shown in Table 5. It can be seen from Table 5 that there is a strong correlation between muscle length and time under the two models; that is, the change trend of the two models is the same. From one-way ANOVA, only the long head of triceps brachii had significant difference. Moreover, if the confidence level is set to 0.01, there is no significant difference between the data obtained by the two models, and the results under the two models show a strong correlation. The above results show that the musculoskeletal model established in this paper can well predict the relationship between muscle length and time in the process of elbow flexion and extension.

Finally, the resultant moment of each muscle in the elbow joint is calculated by the model, and the flexion direction is set as the positive direction. As shown in Figure 11, the comparison diagram of the muscle resultant torque of the elbow joint under the three models is shown, in which the red line represents the torque calculated by the improved musculoskeletal model, the black line represents the torque calculated by OpenSim, and the blue line represents the torque calculated by the common double-muscle musculoskeletal model. The muscle activation degree used in these models is exported through OpenSim. It can be seen from the figure that the torque-time curve calculated by OpenSim and the improved musculoskeletal model is consistent. Compared with the commonly used double-muscle musculoskeletal model, the improved musculoskeletal model proposed in this paper has a better prediction effect.

To verify whether the improved musculoskeletal model and OpenSim model can be regarded as equivalent furtherly, the resultant moments predicted by the two models are analyzed.  Table 6 shows the analysis results. It can be seen from the table that the resultant moment-time relationship calculated by the two models shows a very strong correlation, and there is no significant difference. Therefore, the musculoskeletal model established in this study can be regarded as equivalent to the model in OpenSim.

As shown in Figure 12, it is the elbow torque distributed among the muscles calculated according to the model in this paper. The elbow joint flexes 90° from 0° and then extends back to 0° (elbow angle *θ* = 45 + 45∗sin(*π*t − *π*/2)).

The black solid line is the resultant moment, which is mainly to help the forearm overcome the gravity movement. Therefore, the resultant moment increases with the elbow flexion (forearm lifting). When the elbow is extended (forearm lowering), the resultant moment decreases gradually.

The green line represents the flexion muscle group, and the red line represents the extensor muscle group. During the flexion process (0-1 s), the long head of biceps brachii contributed the most important flexion torque. The initial flexion moment is provided by passive force of the biceps brachii muscle fibers. At the initial stage, the triceps muscle torque is small, mainly to help to maintain the stability of elbow movement. When the angle of the elbow joint approaches 90°, the length of the long head of the triceps brachii exceeds the resting length, resulting in the muscle fibers' passive force. Therefore, the muscle torque of the long head of the triceps brachii becomes larger.

During extension (1-2 s), the muscle torque of the flexion muscle group gradually decreases with the extension of elbow joint. The muscle torque of the long head of triceps brachii also decreased gradually. The main reason is that the long head of triceps brachii is gradually reduced during extension. Although the active force increases, the overall muscle torque decreases due to the small degree of muscle activation.

In the whole movement process, because gravity and flexion muscle force are antagonistic to each other, it can be clearly seen that flexion muscle group plays a major role in joint flexion and extension, while the extension torque of triceps brachii is relatively small. The musculoskeletal model established in this paper can explain the changes of equivalent muscle torque of main muscles during elbow flexion and extension.

## 5. Conclusion

For the estimation of elbow muscle torque, this paper presents an improved elbow musculoskeletal model. In the model, the biceps and triceps are divided into individual two and three muscles, and the brachialis is added as the flexor, which is different from the traditional elbow double-muscle musculoskeletal model. At the same time, the structure of the humeral trochlear is considered. The improved model has more complete muscle quantity, and the geometric model is more in line with the physiological structure. The simulation results show that the model can well predict the muscle torque of the elbow joint. Compared with the elbow muscle torque obtained by OpenSim simulation, the Pearson correlation coefficient shows a very strong correlation, and the one-way ANOVA shows no significant difference between the two models, indicating that the improved elbow neuromusculoskeletal model established in this paper can well predict the elbow muscle torque. However, there are still some problems. Firstly, this paper does not consider the influence of double-joint muscles on elbow muscle torque prediction during shoulder movement. At the same time, although increasing the number of muscles can improve the accuracy of muscle torque prediction, it makes the prediction and parameter optimization process more complex and time-consuming. Therefore, the model established in this paper is not suitable for real-time control of rehabilitation robots or exoskeletons, but it is suitable for evaluating the training effect and guiding the design of rehabilitation robots and prostheses when there is a need to estimate muscle elbow torque.

## Figures and Tables

**Figure 1:** The improved Hill musculotendon model.

**Figure 2:** Calculation flow of the Hill musculotendon model.

**Figure 3:** Comparison of elbow musculoskeletal models.

**Figure 4:** Sagittal view of the humeral ulnar joint during flexion.

**Figure 5:** Schematic diagram of the improved musculoskeletal model of the elbow joint established in this paper.

**Figure 6:** Elbow muscle torque prediction workflow.

**Figure 7:** Planned elbow angle change.

**Figure 8:** The related muscle activation obtained by OpenSim.

**Figure 9:** Muscle force and time relationship under the two models.

**Figure 10:** Muscle length and time relationship under two models.

**Figure 11:** Comparative diagram of elbow joint muscle resultant torque predicted by three models.

**Figure 12:** Elbow torque distributed among the muscles calculated according to the model in this paper.

**Table 1:** Values of formula parameters in the musculoskeletal model in this paper.

Item	Name	Value
Shape coefficient of *f*_l_	*γ*	0.5
Curve parameters of *f*_v_	*A*_s_	0.25
Maximum muscle force during muscle fiber elongation	*f*_M_	1.8
Normalized muscle fiber maximum contraction velocity	*v*_n_	8*l_mopt_*
Shape parameters of passive force curve	*k* ^PE^	4
Maximum passive tension strain	*ε*_0_^M^	0.5
Muscle force arm shape parameters	*k*_s_	0.004

**Table 2:** Relevant personalized parameters used in this paper.

Name	*l*_mopt_ (m)	*l*_topt_ (m)	*F*_0_ (N)	*φ*_0_ (°)
Long head of biceps brachii	0.116	0.272	624.3	0
Short head of biceps brachii	0.132	0.192	435.6	0
Brachialis	0.086	0.054	987.3	0
Long head of triceps brachii	0.134	0.143	798.5	12
Lateral head of triceps brachii	0.114	0.091	624.3	9
Medial head of triceps brachii	0.114	0.098	624.3	9

**Table 3:** Spatial position of starting and ending points of flexion muscles.

Name	Starting point	End point	*l*_0_ (m)
Long head of biceps brachii	(0.023, 0, 0.115)	(0.007, 0, -0.047)	0.263
Short head of biceps brachii	(0.023, 0, 0.115)	(0.007, 0, -0.047)	0.178
Brachialis	(0.008, 0, 0.115)	(0.007, 0, -0.023)	0.010

**Table 4:** Comparative analysis results of muscle force-time relationship.

Muscle	Pearson correlation coefficient			One-way ANOVA (*α* = 0.05)			
	OpenSim	Improved model	Result	*F*	*P* value	*F*-crit	Result
Biceps long	1	0.993	ESC	2.664	0.103	3.865	NSD
Biceps short	1	0.975	ESC	16.08	7.21*E*-05	3.865	ESD
Brachialis	1	0.943	ESC	9.468	2.23*E*-3	3.865	ESD
Triceps long	1	0.999	ESC	2.508	0.114	3.865	NSD
Triceps lateral	1	0.995	ESC	0.149	0.903	3.865	NSD
Triceps medial	1	0.969	ESC	38.325	1.5*E*-3	3.865	ESD

**Table 5:** Comparative analysis results of muscle length-time relationship.

Muscle	Pearson correlation coefficient			One-way ANOVA (*α* = 0.05)			
	OpenSim	Improved model	Result	*F*	*P* value	*F*-crit	Result
Biceps long	1	0.999	ESC	0.028	0.876	3.865	NSD
Biceps short	1	0.999	ESC	0.948	0.331	3.865	NSD
Brachialis	1	0.998	ESC	0.235	0.628	3.865	NSD
Triceps long	1	0.999	ESC	5.887	0.016	3.865	ESD
Triceps lateral	1	0.999	ESC	0.003	0.953	3.865	NSD
Triceps medial	1	0.999	ESC	1.978	0.160	3.865	NSD

**Table 6:** Comparative analysis of the predicted resultant moment-time relationship.

Pearson correlation coefficient			One-way ANOVA (*α* = 0.05)			
OpenSim	Improved model	Result	*F*	*P* value	*F*-crit	Result
1	0.970	ESC	1.390	0.239	3.865	NSD

## Data Availability

The data are made available through the corresponding authors' emails.
